# Evaluation of the Effectiveness of Artificial Neural Network Based on Correcting Scoliosis and Improving Spinal Health in University Students

This article has been retracted.

**DOI:** 10.1155/2022/2092034

**Published:** 2022-02-10

**Authors:** Jiefu Peng

**Affiliations:** Department of General Education, Southern Medical University, Guangzhou 510510, China

## Abstract

In recent years, spinal disorders, spinal deformities, and scoliosis have become more frequent, especially chronic systemic inflammatory diseases, such as early-onset scoliosis, idiopathic scoliosis, and ankylosis spondylitis, which have unknown causes, insidious onset, and progressive development, resulting in irreversible spinal joint deformities and stiffness at advanced stages and high disability rates. As one of the traditional Chinese health and fitness qigong exercises, Taijiquan has the effect of strengthening the waist and kidneys, sparing the tendons and softening the body, unblocking the meridians, unblocking the qi and blood, and strengthening the body and increasing intelligence. To this end, this paper proposes a data enhancement method that uses the spine line as the control curve to deform the human contours, drawing on the moving least squares deformation method to fit a variety of scoliosis cases and increase the diversity of the dataset, thereby improving the generalisation capability of the network. The colour map and depth map information are then integrated using a four-channel method and a dual feature extraction network structure to improve the accuracy of segmentation.

## 1. Introduction

Prolonged sitting posture can bring static damage to the spine, especially prostration in the seat and various poor sitting postures, which can easily cause asymmetry and twisting and stretching of the muscles around the spine, making the spinal system unbalanced and thus causing discomfort to the shoulder, neck, and back [1]. The longer the setting time, the higher the proportion of cervical spondylitis, lumbar spondylitis, and frozen shoulder [2]. Other studies have found that spinal curvature and activity are related to physical activity and that excessive physical activity or incorrect posture during mirror physical activity may have a corresponding effect on the sagittal curvature and activity of the thoracolumbar segment of the spine, causing spinal curvature and mobility abnormalities, resulting in injury to the spine and even disease [3]. Chronic low back pain is associated with changes in the structural function of the lumbar muscles, decreased muscle strength, and structural degeneration of the lumbar spine, which can lead to low spinal stability, trunk muscle strength, explosive strength of the extensor muscles, and imbalances in flexion and extension muscle strength, resulting in varying degrees of degenerative lesions in the morphology and structure of the lumbar segment of the spine and surrounding tissues [4]. In addition, long-term muscle fatigue can also cause calcification of the musculoligamentous junction with the bone, resulting in diseases such as cervical and lumbar spine osteomalacia [5]. Therefore, prolonged poor body posture during bone growth and development or in daily life can lead to tissue damage that can restrict spinal movement and even compromise spinal health. For example, [6] reported that prolonged forward head tilt can lead to shortening of tension in the cephalitis, superior trapezius and sternocleidomastoid muscles, and weakness of the middle trapezius bundle, affecting the contractile activity of the muscle length.

Young people who have just entered university develop sedentary habits due to excessive study pressure or addiction to games in high school, and long-term unreasonable sitting posture leads to different degrees of damage to the spine, causing abnormal curvature of the spine and eventually leading to various spinal disorders.

Taijiquan is one of the oldest, most widespread, and most influential fitness and qigong techniques in China, and nowadays it has formed an independent and complete set of fitness methods. Because it is an aerobic endurance exercise with few movements, is easy to learn, and has moderate intensity, it is not only favoured by the middle-aged and elderly but also considered an important physical therapy tool for health and disease prevention in Chinese medicine [7]. Traditional Chinese medicine believes that technique has the function of softening the tendons and bones, nourishing the qi and strengthening the strong, moving the qi and activating the blood, and harmonising the five organs and six internal organs.

The human spine is made up of a number of vertebrae combined by ligaments, intervertebral discs, and bone joints. In the sagittal plane, the spine has an anteriorly convex cervical, a posteriorly convex thoracic, an anteriorly convex lumbar, and a posteriorly convex sacral form and is divided into three segments: cervical, thoracic, and lumbar according to their mobility [8]. The different segments of the vertebrae are linked to bony links so that the body can freely flex, extend, rotate, and turn sideways, with the assistance of muscles, ligaments, and other body tissues to ensure the stability of the spine and a greater range of movement. The nerve, muscles, ligaments, and other tissues attached to the spine and its surroundings are therefore essential for the maintenance of normal spinal movement and protection of the spine [9].

Tahitian is unique in its effectiveness in preventing abnormalities in spinal mobility. (1) Through the rotational stretching of the spine, the nerve impulses of the tissues and organs are raised, skeletal muscle stagnation is reduced, the muscles on both sides of the spine are strengthened, and the body posture is corrected. For example, in the first four postures, the upward and downward stretching and rotation of the two hands on the sky, the left and right open bow, the one-handed symmetrical pressing and lifting, and the rotating back look not only lengthen the muscles, ligaments, and joint tissues around the joints of the trunk and upper limbs but also exercise the small joints and muscles between the vertebrae in the spine, thus enhancing the flexibility and stability of the spine, and increasing the contraction force of the muscles involved in movement around the neck and shoulder joints, as well as the range of neck movement. It also increases the contraction force of the muscles involved around the neck and shoulder joints, as well as the range of neck movement. It has an important role in correcting poor posture, improving blood circulation in the neck and brain, and relieving central nervous system fatigue [10]. It can effectively prevent and treat scoliosis, cervical spondylosis, rotational misalignment of the thoracic spine, and lumbar back strain, as well as correcting small joint misalignments, improving neck mobility, and changing the physiological curvature of the spine [11].

## 2. Related Work

In recent years, research into the rehabilitation of CNLBP in Taijiquan has mainly used experimental interventions to assess patients' signs using scales, such as the Visual Analogue Pain Scale (VAS), the Questionnaire of Functional Impairment (Qswestry), and the JOA, and experimental equipment or systems such as the Surface Electromyography Tester and the Spinal Mouse Spine Function Tester are also gradually being used. In addition, experimental devices or systems, such as the surface electromyography tester and the Spinal Mouse spinal function tester, have been gradually applied to this field of study. By recording and analysing changes in the surface EMG signal characteristics, subjective pain sensation, and core muscle potential energy in patients with chronic lower back pain, it was concluded that regular tactical exercises were more effective than core stability training in engaging the superficial muscle motor units, improving the imbalance of the rectus abdominis, external abdominal oblique, and vertical spinal muscles, improving static endurance of the low back muscles, and also improving the strength of the patient's low back muscles to some extent [12]. Reference [13] used an event-related potential (ERP) study to investigate the mechanism of tactician's effect on the cognitive function of patients with chronic lower back pain and concluded that tactician training could improve pain perception and reduce pain sensitivity in patients with chronic lower back pain. Reference [14] concluded that tai chi exercises could increase the stability of the stride of patients with chronic lower back pain and strengthen the muscles of the lower limbs; it could improve the flexion and extension of the hip and ankle joints as well as the range of motion of the three joints of the lower limbs. The effects of taxation “flashing through the dark” on the function of the lumbosacral multitudes muscles in patients with chronic nonspecific lower back pain were observed by using VAS visual analogue scoring, surface electromyography, and isometric muscle strength testing [15].

In conclusion, regular tactician practice appears to be more effective in the rehabilitation of patients with CNLBP than core stability training, walking, or other exercise therapies alone [16]. Long-term regular tactician exercise increases the strength of the patient's low back muscles, reduces sensitivity to low back pain, improves gait patterns in a coordinated manner, and improves spinal stability. Taijiquan is mainly used to reduce the subjective perception of pain in CNLBP patients and improve their ability to perform daily activities through internal conditioning and external exercise, thus achieving a reduction in symptoms and a gradual recovery of health.

## 3. Causes of Scoliosis

Scoliosis is a spinal deformity growth disorder commonly seen in adolescents and is characterised by fixed lateral curvature and rotational deformity of the spine. According to criteria established by the Scoliosis Research Society, structural scoliosis is defined when the positive plane curve observed in the anterior posterior plane is greater than 10° [17]. Scoliosis can be extremely harmful to the human body, as it not only affects the normal development of the skeleton, causing imbalance of forces on both sides of the spine and back pain but also may cause compression of the spinal cord, thoracic cavity, and abdominal cavity, seriously affecting the function of various body systems and even the life of the patient [18].

Currently scoliosis is mainly diagnosed using X-rays. The severity of scoliosis is assessed by taking forward and lateral X-rays of the entire spine while the patient is standing, and then calculating the size of the Cobb angle in the image [19]. Current treatments for scoliosis include nonsurgical treatment based on thoracolumbosacral orthoses and surgical treatment based on spinal fusion [20], but each of these treatment options requires an X-ray to be obtained every 6 to 12 months and the magnitude of the curve to be assessed continuously using the Cobb angle and other standard measurements. Because X-rays are radioactive, multiple exposures can be damaging to the body and are not conducive to continuous assessment of the spine curve, and it has been shown that female patients with scoliosis in childhood or adolescence have an increased risk of breast cancer when regularly exposed to low levels of ionising radiation [21]. In addition, X-rays are not useful for the measurement of rotational deformation of the spine in the horizontal plane, as shown in Figure 1.

## 4. Programme of This Paper

### 4.1. Control Point Based on Moving Least Squares Deformation

Considering the deformation of an image as a deformation function *f*, let the image before the deformation be *X* and the image after the deformation be *Y*; then, the process of deformation of the image can be described as

(1) $$\begin{array}{c} y=f\left(x\right). \end{array}$$

Let *s* be the set of control points before the image deformation and *d* the set of control points after the deformation. According to the principle of least squares, the mapping function *f* for each pixel *x* in the image *X* before the deformation needs to be minimized in

(2) $$\begin{array}{c} C=\sum_{i}w_{i}{\left|f\left(s_{i}\right)-d_{\text{i}}\right|}^{2}, \end{array}$$

where *w*_*i*_ is the weight and the expression is

(3) $$\begin{array}{c} w_{i}=\frac{1}{{\left|s_{i}-x\right|}^{2\alpha }}, \end{array}$$

where *α* is a factor regulating the effect of deformation.

The deformation function *f* includes both linear and translational transformations so that *f* can be expressed in the following form:

(4) $$\begin{array}{c} f\left(x\right)=xM+T, \end{array}$$

where *M* is the linearly transformed 2 × 2 matrix and *T* is the translational 1 × 2 matrix.

Bringing (4) into (3) to find the minimum, that is, solving for the derivative *dC*/*dT*=*d*(∑_*i*_*w*_*i*_|*s*_*i*_*M*+*T* − *d*_*i*_|^2^)/*dT*=0, gives

(5) $$\begin{array}{c} T=\frac{\sum w_{i}d_{i}}{\sum_{i}w_{i}}-\frac{\sum_{i}w_{i}s_{i}}{\sum_{i}w_{i}}M. \end{array}$$

The general form of the deformation function *f* is obtained from (5):

(6) $$\begin{array}{c} f\left(x\right)=\left(x-\frac{\sum_{i}w_{i}s_{i}}{\sum_{i}w_{i}}\right)M+\frac{\sum w_{i}w_{i}}{\sum_{i}w_{i}}. \end{array}$$

By bringing (6) into (2), (2) can become

(7) $$\begin{array}{c} C=\sum_{i}w_{i}{\left|\left(s_{i}-\frac{\sum_{i}w_{i}s_{i}}{\sum_{i}w_{i}}\right)M-\left(d_{i}-\frac{\sum_{i}w_{i}d_{i}}{\sum_{i}w_{i}}\right)\right|}^{2}. \end{array}$$

Let, $s_{x}=\sum_{i}w_{i}s_{i}/\sum_{i}w_{i},d_{x}=\sum_{i}w_{i}d_{i}/\sum_{i}w_{i},\hat{s}=s-s_{x},\hat{d}=d-d_{*}$; then, *C* can be rewritten as

(8) $$\begin{array}{c} C=\sum_{i}w_{i}{\left|\hat{s}M-\hat{d}\right|}^{2}. \end{array}$$

As can be seen from (8), *f* is mainly determined by the linear transformation matrix *M*, which contains the various operations of the affine transformation, including scaling, rotation, and misalignment. Different combinations of the various operations in the affine transform lead to three image deformation algorithms: the affine transform, the similarity transformation, and the rigid transformation, which are shown in Figure 2 for the cartoon character.

### 4.2. Multiview Learning Based on Deep Information

In automatic mechanical scanning, depth map data is usually used only to obtain the three-dimensional spatial coordinates by which the mechanical device performs accurate scanning, without processing the depth map information during the path planning phase [22]. However, the body contours can also be distinguished in the depth map, and there are obvious depth variations in the spine region, so the relationship between the spine region and the body contours can be analysed from a depth perspective, and the obvious boundaries of the body contours in the depth map and the depth variations in the spine region can be added to the network as a learned feature for training to obtain better segmentation results.

In order to verify the information validity of the depth images, this paper has done the results based on the DeepLab network using only the depth images as training data, and the standard errors on the validation set are shown in Table 1.

Table 1 shows that the depth image contains information about the spine region of the human body and that the convolutional neural network can extract this feature from the image and make the correct segmentation decision.

In this paper, two methods of introducing depth information are used: one method is the four-channel method, in which the depth information is used as an input channel and fed into the feature extraction network of the full convolutional network together with the three channels of RGB [23]; the other method is to process the depth image as a separate image, build a special convolutional network to learn the features of the depth map, and then through certain processing, the depth information of the feature map of the depth information is then fused with the feature map of the colour information through certain processing to jointly influence the final segmentation effect.

#### 4.2.1. Four-Channel Method

This method treats the depth map as an input channel and normalizes the depth value to [0, 1] and then, together with the three RGB channels, forms the RGB-D four input channels into the convolutional neural network to obtain the segmentation result. This is a relatively simple and effective method in which the network built in the previous section does not need to be changed much, but only one channel is added to the input layer, as shown in Figure 3.

However, this method has some obvious disadvantages: in the RGB channel, there is a significant difference between the brightness of the human skin and the surrounding background; that is, the values of the three RGB channels in the background differ significantly from the values of the human body area, while the spine area has shadow characteristics due to its concave and convex characteristics, usually showing low brightness in the concave shadow areas and high brightness in the raised areas, and the difference in the values of the three RGB channels is also relative. The difference in values between the three RGB channels is also noticeable. In the depth map, the difference between the spine and the rest of the body is relatively small, and the body and the background are in a strict depth progression, so the data distribution of the depth map is not consistent with that of the colour map, and there is a certain semantic gap, which has an impact on the learning of the network [24].

#### 4.2.2. Dual Feature Extraction Network Method

In order to solve the semantic gap between depth information and RGB information, this paper builds a new network model based on the full convolutional network, using the method of feature extraction and segmentation for colour images and depth images, respectively, and then fusing the segmentation results, the network model is shown in Figure 4.

Where the network performs feature extraction separately for colour and depth images, the feature extraction part is as deep, first using a convolution kernel size of 7 × 7, the number of 64 convolution layers and a maximum pooling layer to reduce the image size, immediately followed by three residual modules in which each module has 3 residual units and each residual unit is the same as the three-layer residual learning unit model. The null convolution module has 16 residual units; each residual unit is similar to the three-layer residual learning unit model, but the number of convolution kernels is changed to 256, 256, and 1024, where the middle convolution layer is set to null convolution with rate = 2. The final layer is the porous pyramid pooling layer, which is used to integrate results from different scales. After completing the independent segmentation of the depth image and the colour image, the segmentation results are integrated using stacking, and finally a convolutional layer with a convolutional kernel size of 3 × 3 and a number of classification categories is used to learn the weights of the two feature maps to obtain the best segmentation results.

The network is trained with colour and depth images for input 1 and input 2, respectively, and a mask for the output. The parameters obtained from training DeepLab with colour images and the parameters obtained from training DeepLab with depth images only are used to initialise the network; otherwise, the network will be too large and difficult to converge.

## 5. Case Studies

A group of students was initially screened in the university physical fitness test, and spinal mobility was measured using a spine measuring device. The subjects were randomly divided equally into an experimental group [20] and a control group [20] in equal proportions of male and female. The experimental group underwent Taijiquan intervention for 3 months; the control group maintained a normal lifestyle without any intervention. The differences in body mass index (BMI), height, and weight between the experimental group and the control group before the intervention were not statistically significant (*P* value >0.05).

The subjects screened were informed of the intent of this experiment and signed an informed consent form to voluntarily participate in the experiment. The study was approved by the Ethics Committee of the university as a provincial project of university students' innovation and entrepreneurship. The subjects were first trained to teach exercise 2 weeks before the intervention in the experimental group, explaining the technical aspects of tactical movements to the subjects and correcting errors. The participants practiced for 3 months, 4 times a week for 1 h, including 5–10 min of preparation, 40–50 min of tactician practice, and 5–10 min of finishing activities; each time, the whole set of movements was practiced 3 times, the individual movements of each form were repeated 3–7 times, and the interval between each tactician exercise was 2–3 min.

After the Taijiquan exercise intervention, the spinal tilt angle of the university students in the experimental group was corrected by 1.70° on average; the anterior-posterior convexity of the spine of the subjects was significantly improved; the left- and right-side curvatures of the cervical spine were increased by 7.30° and 7.90°, respectively, and the left- and right-side curvatures of the thoracic spine were increased by 5.35° and 7.00°, respectively (*P* values <0.05); the left- and right-side curvatures of the lumbar spine were not significantly improved, but there were more significant changes compared to the control group. The lumbar left and right lateral bending did not improve significantly, but there was a more significant change compared to the control group. The anterior and posterior flexion and extension of the cervical spine improved significantly, with an increase in flexion and extension of 9.25° and 8.00°, respectively; the anterior and posterior flexion and extension of the thoracic spine improved significantly, with an increase in flexion and extension of 8.90° and 11.35°, respectively; the anterior flexion and extension of the lumbar spine improved significantly, with an increase in anterior flexion of 6.45° (all *P* values <0.05), and the posterior extension of the lumbar spine did not change significantly relative to the pretest but did change significantly relative to the control group. There was no significant change in lumbar posterior extension compared to before the experiment, but there was a significant change compared to the control group [25]. The rotational capacity of the spine was improved by the tactician intervention, with an increase of 5.40° and 8.70° in the left and right rotation of the cervical spine, respectively, and an increase of 5.60° in the left rotation of the thoracic spine (all *P* values <0.05); there was no significant change in the right rotation of the thoracic spine, but there was a significant change in the right rotation of the thoracic spine compared to the control group. Values were <0.05. The balance of the spine was significantly altered by the tactician intervention, with the cervical, thoracic, and lumbar spine balance improving by 0.50°, 0.70°, and 0.45°, respectively (all *P* values <0.05). See Table 2.

## 6. Analysis of Model Results

Similarly, in this section, the standard errors between the two curves defined for the improved algorithms are quantitatively compared using the DeepLab network with three channels of input, the DeepLab network with four channels of input, and the dual feature extraction network, respectively. The mean standard deviation before data augmentation represents the standard error of the validation set segmentation results against the manually drawn curves after training with a training set that does not incorporate moving least squares deformation images, the mean standard deviation after data augmentation represents the standard error of the validation set segmentation results against the manually drawn curves after training with a training set that incorporates moving least squares deformation images, and the mean standard deviation under the improved postprocessing algorithm represents the standard error of the scan curves obtained using the human contour and curve fitting based on the standard error of the scanned curves obtained after postprocessing versus the manually drawn curves.

As can be seen from Table 3, there was little reduction in segmentation error before and after the use of data augmentation, which was due to the small number of back maps collected from scoliosis patients, which did not reflect a significant segmentation effect on scoliosis patients. After adding depth information for training, the segmentation accuracy was significantly improved and the network missegmentation was significantly reduced. Finally, due to the high number of missegmentations in the direct segmentation of colour maps, the error was significantly reduced using the improved postprocessing algorithm, while in the combined learning of colour and depth information, there were fewer missegmentations and the use of the improved postprocessing algorithm was not as effective but still reduced the error by curve-fitting tandem segmentation of broken regions.

## 7. Analysis of Chen's Taijiquan for Correction of Spinal Curvature

Methods were as follows. A 6-month experiment on the correction of spinal curvature was conducted on 40 university students using Chen's Taijiquan exercises combined with physical rehabilitation. Results were the following. The average reduction of anterior neck curve was 0.96 cm (*P* < 0.05), 12 university students with excessive anterior neck curve returned to normal range, the average reduction of anterior lumbar curve was 0.25 cm (*P* < 0.05), and 4 university students with excessive anterior curve corrected to normal range, and the average increase of lung capacity was 75 ml. The combination of Chen's tactician practice and physical rehabilitation correction training had a significant effect on college students' spinal curvature and improved lung capacity. The result is shown in Table 4.

The adult spine, when viewed from the side, is curved in an “*S*” shape from top to bottom. These are the anterior cervical curve, the posterior thoracic curve, the anterior lumbar curve, and the posterior sacral curve. This physiological anterior curvature is often exacerbated by chronic poor posture, heavy study loads, nearsightedness, unilateral weight bearing, lack of physical activity, frailty, or malnutrition and even exceeds the normal range, resulting in severe deformation of the spine. Abnormal spinal curvature not only affects the beauty of the body but also hinders the normal development and function of internal organs, reduces lung capacity, and decreases the flexibility of the spine. As shown in Figure 5, the effect of different times of technician training, due to the loss of balance in the point of action of the force, people with abnormal spinal curvature are also prone to fatigue after study or work and, in serious cases, even to varying degrees of loss of labour [26]. At the same time, excessive anterior neck flexion is often accompanied by an increase in posterior thoracic flexion, which is the result of a combination of anterior neck flexion and posterior thoracic flexion.

As shown in Figure 6, the results of the 6-month Chen's Taijiquan practice combined with physical rehabilitation training for 40 university students with excessive anterior neck curvature showed that the average anterior neck curvature decreased from 6.35 cm to 5.26 cm before the experiment; although the mean value after the experiment was still higher than the normal range, 12 of the 40 students with excessive spinal curvature returned to the normal range, accounting for 30% of the total sample. This represents 30% of the total sample. The mean value of the anterior lumbar curve before the experiment was 3.98 cm, which was within the normal range of 3.0–5.0 cm. The variation of the samples ranged from 2.5 to 6.1 cm, with only four cases of anterior lumbar curve exceeding the normal range of 5.0 cm, accounting for 10% of the total sample. However, after the experiment, the mean value of anterior lumbar flexion changed to 3.37 cm. *P* < 0.05, which was statistically significant before and after the experiment. Four samples with anterior convexity were also fully adjusted to within the normal range. This again suggests that Chen's Taijiquan practice combined with physical rehabilitation correction training is also effective in correcting anterior lumbar curvature [27].

As showed in Figure 7, 6 months of Chen's Taijiquan practice combined with sport rehabilitation correction training not only had a good corrective effect on the anterior cervical curvature but also had a significant improvement on the anterior lumbar curvature and increased lung capacity. During the 6 months of training, no negative effects were observed. Chen's Taijiquan is a traditional Chinese martial art, and its “virtual collar and top strength” is conducive to straightening the cervical vertebrae, relaxing the neck muscles, coordinating and balancing them, restoring the spinal cord, blood vessels, and trachea to their normal position, and making the whole spinal column upward; “chest and back extraction” can increase the volume of the thoracic cavity, increase lung capacity, make breathing deeper and smoother, and at the same time facilitate the movement of the diaphragm; “loosening the hips and wrapping the buttocks, making the door of life convex” is conducive to the relaxation of the hip sockets on both sides and the downward sagging of the hip muscles, so that the anterior curvature of the lumbar vertebrae is weakened or disappears. Combined with “qi sinking into the dantian,” the whole spine is pulled down. In general, pulling up and pulling down is a manifestation of modern medical “traction” in tactician, which is one of the most effective means of modern medicine for spinal deformation. Physical rehabilitation training is a method of exercise for the cervical and thoracic spine, which allows the muscles and ligaments attached to the spine to be properly exercised, such as traction on the anterior longitudinal ligament [28], which stretches it and helps to reduce the curvature of the posterior thoracic curve; strengthening the back muscles and improving their tension can reduce the posterior thoracic curve and anterior cervical curve, ultimately achieving the goal of complete rehabilitation [29].

## 8. Conclusions

The spinal column is damaged to varying degrees due to unreasonable sitting posture. Taijiquan, as one of the traditional Chinese health and fitness qigong exercises, has the effects of strengthening the waist and kidney, sparing the tendons and softening the body, unblocking the meridians, unblocking the qi and blood, and strengthening the body and increasing the intelligence. This paper proposes a data enhancement method to deform the human contours using the spine line as the control curve by borrowing the moving least squares deformation method to fit a variety of scoliosis cases and increase the diversity of the data set, thus improving the generalisation ability of the network. The aim of this study is to investigate the changes in spinal mobility after the experiment through the intervention of tai chi exercise on the spinal mobility of university students and to provide a basis and method for the prevention and treatment of promoting the spinal health of university students.

## Figures and Tables

**Figure 1:** Radiographs of scoliosis and calculation of Cobb's angle. (a) X-ray diagram of scoliosis and (b) calculation diagram of Cobb's angle.

**Figure 2:** Schematic diagram of the affine and similar and rigid transformations of a cartoon character. (a) Original picture, (b) affine transformation, and (c) similarity transformation.

**Figure 3:** Schematic diagram of the four-channel method.

**Figure 4:** Schematic diagram of the DeepLab-based dual feature extraction network structure.

**Figure 5:** Effect of taijiquan training at different times.

**Figure 6:** Correction errors for different methods.

**Figure 7:** Different exercise rehabilitation effects.

**Table 1:** Mean standard errors using depth data.

Network model	Mean standard error
DeepLab	8.21007

**Table 2:** Pre- and postexperimental comparison between the experimental and control groups of university students on various indicators of spinal mobility ($\bar{x}\pm s$).

Index	Experimental group (*n* = 20)				Control group (*n* = 20)			
	Before experiment	After the experiment	*T*	*P*	Before experiment	After the experiment	*T*	*P*
ATI	4.8 ± 1.88	3.10 ± 1.21	3.40	0	4.8 ± 1.88	5.15 ± 1.69	−0.62	0.54
Kyphosis	22.40 ± 6.23	23.30 ± 3.81	−2.87	0.6	22.15 ± 6.07	22.10 ± 7.12	0.24	0.98
Left cervical curvature	41.65 ± 8.41	48.95 ± 7.65	−2.87	0.01	41.08 ± 7.40	42.30 ± 5.87	−0.25	0.80
Right cervical curvature	41.45 ± 9.23	49.35 ± 8.02	−2.82	0.01	42.25 ± 10.31	44.70 ± 7.02	−0.88	0.39
Left thoracic curvature	40.45 ± 9.28	45.80 ± 4.57	−2.34	0.03	38.35 ± 9.17	39.55 ± 4.87	−0.52	0.61
Right thoracic curvature	36.90 ± 6.71	43.90 ± 3.61	−4.11	0	37.35 ± 6.41	37.45 ± 6.01	−0.05	0.96
Left lumbar curvature	20.85 ± 5.30	26.35 ± 5.28	−1.67	.01	20.58 ± 5.26	19.85 ± 4.12	0.67	0.51
Lumbar right curvature	20.65 ± 6.00	24.35 ± 5.61	−2.01	0.05	20.60 ± 4.39	20.60 ± 8.44	0.77	0.44
Left cervical rotation	66.55 ± 8.79	71.95 ± 7.06	−2.14	0.04	67.15 ± 8.76	67.95 ± 10.79	−0.26	0.80
Right cervical rotation	66.80 ± 11.72	75.50 ± 9.16	−2.62	0.01	67.95 ± 12.11	68.35 ± 11.52	−0.11	0.92
Thoracic left rotation	37.10 ± 6.33	42.70 ± 6.25	−2.82	0.01	35.55 ± 6.98	37.80 ± 8.28	−0.95	0.36
Thoracic right rotation	35.25 ± 10.09	40.75 ± 7.15	−1.99	0.05	34.20 ± 9.05	35.85 ± 8.91	−0.85	0.57
Lumbar left rotation	18.50 ± 6.30	22.40 ± 5.86	−1.67	0.06	18.10 ± 6.44	18.30 ± 4.45	−0.11	0.91
Lumbar right rotation	18.85 ± 6.87	20.35 ± 3.79	−0.68	0.50	19.10 ± 5.66	20.00 ± 4.31	−0.57	0.58
Cervical balance	0.85 ± 0.99	0.35 ± 0.58	−0.19	0.06	0.70 ± 0.86	0.75 ± 0.85	−0.18	0.86
Thoracic balance	0.95 ± 0.83	0.25 ± 0.44	3.34	0	0.85 ± 0.81	0.75 ± 0.64	0.43	0.67
Lumbar spine balance	1.10 ± 0.79	0.65 ± 0.49	2.17	0.04	1.15 ± 1.09	1.40 ± 0.55	0.18	0.89

**Table 3:** Mean standard errors of the different models.

Network model	Mean standard error before data enhancement	Mean standard error after data enhancement	Average standard error under improved postprocessing algorithm
Three-channel model	7.57703	6.13261	4.95387
Four-channel model	4.2971	3.98792	3.66854
Double feature extraction network model	4.12587	3.98753	3.58297

**Table 4:** Comparison before and after the experiment (example).

	*n*	Anterior cervical curvature (CM)	Lumbar lordosis (CM)	Vital capacity (mmHg)
Before the experiment	40	6.32 ± 0 72	3.98 ± 0.97	—
After the experiment	40	5.26 ± 0.74	3.37 ± 0.18	—
Difference	40	−0.96 ± 0.82	−0.25 ± 0.49	75 ± 36.5

## Data Availability

The datasets used during the current study are available from the corresponding author on reasonable request.
